# Shear Wave Elastography-Assisted Ultrasound Breast Image Analysis and Identification of Abnormal Data

**DOI:** 10.1155/2022/5499354

**Published:** 2022-01-07

**Authors:** Caoxin Yan, Zhiyan Luo, Zimei Lin, Huilin He, Yunkai Luo, Jian Chen

**Affiliations:** ^1^Department of Ultrasound in Medicine, The Fourth Affiliated Hospital of Zhejiang University School of Medicine, Yiwu, Zhejiang 322000, China; ^2^Department of Ultrasound in Medicine, The Second Affiliated Hospital Zhejiang University School of Medicine, Hangzhou, Zhejiang 310009, China

## Abstract

In this paper, shear wave elastography was used to study and analyze the images of the breast in-depth and identify the abnormal image data. Sixty breast lesions were evaluated, and quantitative metrics were reproducible in the static and dynamic modes of shear wave elastography with a higher interobserver agreement in dynamic qualitative metrics than in the static mode. There were no statistically significant differences between the two modes of imaging in quantitative metrics, and quantitative metrics were more effective than qualitative metrics. Postoperative immunohistochemical expression of ER, PR, HER-2, Ki-67, molecular typing, pathological type, histological grading, and axillary lymph node status of breast cancer was obtained based on pathological results. The correlation between mass size, patient age, and WiMAX values of breast cancer masses was analyzed using Pearson correlation, and the differences in SWVmax values of breast cancer masses between different expressions of immunohistochemical parameters ER, PR, HER-2, Ki-67, and axillary lymph node status were compared using tests. The variables with correlations and differences were included in the multiple linear regression analysis to assess the factors influencing the SWVmax values. The performance of TDPM, SPM, and TSPM was compared using PVA body models with different freeze-thaw cycles. The results showed that TSPM performed better than SPM in general, and TDPM showed excellent performance because of high temporal resolution and low random error, especially when the number of freeze-thaw cycles increased and the hardness of the PVA body mold increased. Measurements at different depths of inhomogeneous body models also showed that the TDPM method was less affected by depth, and the results were more stable. Finally, the reliability of the shear wave velocity (SWS) measured by the TDPM and SPM methods was investigated using porcine ligament tissue, and the results showed that the mean values of SWS goodness of fit for TDPM and SPM were 0.94 and 0.87, respectively, and the estimated elastic modulus of TDPM was very close to the mechanical test results.

## 1. Introduction

The mammary glands are located on the surface of the chest wall at the level of the second to sixth ribs between the subcutaneous fascia and the fascia of the pectoralis muscle, and they are symmetrical from left to right. The mammary glands consist of 15–20 lobes arranged in a radial pattern with the nipple as the center, and the lobes are composed of lobules, which, in turn, are composed of each branch of the milk duct and its associated alveoli. The milk duct branches begin in the peripheral ducts and merge in a “two-and-one” fashion from the lower ducts to the higher ducts, ending in the milk-transmitting sinus. Most peripheral ducts, terminal ducts, and the surrounding alveolar tissue form the basic unit of the breast tissue, the terminal ductal lobule, which is the site of most breast diseases [1]. Intramammary lumps are a common clinical manifestation of breast disease mostly because of benign conditions such as fibroadenomas and cysts. However, in recent years, the incidence of breast cancer (BC) has been increasing year by year, ranking first among female malignant tumors. Although the prevalence of breast cancer in China is lower than that in Europe and the United States, the statistics are still not optimistic as Chinese women account for 12.2% of the newly diagnosed breast cancer patients worldwide each year. The trend is younger, which is an important cause of premature death in women and brings a heavy burden to families and society, making it a major public health problem [2]. Define the labeled breast tumor image data set in the source domain, and define the unlabeled target breast tumor image data set to be classified as the target domain, which, respectively, represent the number of samples in the source domain and the target domain. However, the mortality rate of breast cancer is decreasing compared to the increasing trend of breast cancer prevalence. At this time, the advantages of conventional ultrasonography (US), which is inexpensive, convenient, and safe without radiation, come to the fore. Conventional 2D ultrasound provides a unique anatomical cross-sectional image of the mass of the surrounding tissues, providing information including mass size, morphology, margins, echogenic pattern, posterior attenuation, and internal calcification, which provides a basis for the detection of breast cancer. The application of Doppler ultrasound is valuable in observing the characteristics of blood flow distribution and hemodynamic features within and around the mass and aids the conventional two-dimensional ultrasound to complete the diagnosis and differential diagnosis. However, it is influenced to some extent by the subjective judgment of the examiner with fair sensitivity and poor specificity [3].

However, as the sonograms of benign breast lesions and breast cancer overlap to a certain extent and the sonograms of breast cancer lesions are complex and variable because of the diversity of their clinicopathological features, conventional color Doppler ultrasonography has some limitations to some extent. Although ultrasound elastography, which generates strain by applying pressure, helps assist diagnosis, it is susceptible to physician subjectivity and manipulation during operation [4]. In contrast, real-time shear wave elastography (SWE), also known as E imaging, is a new quantitative ultrasound elastography technique that obtains elastic modulus values by quantitatively detecting the actual stiffness of the breast masses, thus providing a more objective and quantitative evaluation of breast lesions. It can overcome interference from the tissues outside the region of interest with high reproducibility. It has advantages in unique diagnostic and differential diagnosis in breast diseases, and thus it can overcome the subjective influence and inherent defects of stress elastography.

However, morphological criteria alone are not sufficient to measure the nature of breast masses. In clinical applications, the same lesions show different hardness values on different machines, probably because different manufacturers apply different imaging principles. The Mindray Reson 7 machine offers both shear wave static and dynamic elastography, where a higher quality image can be obtained on static mode elastography. However, in dynamic mode elastography, three levels of frame rate can be selected (0.4, 0.7, and 1.0 frames/sec) to choose the best quality one among multiple consecutive images. It may be more advantageous for areas affected by cardiac motion advantage. Little research has been done on the superiority of these two modes of elastography for the diagnosis of breast lesions. The purpose of this section is to evaluate the interobserver agreement between the qualitative and quantitative indices of static and dynamic imaging modalities and the diagnostic efficacy of the same for breast lesions and to compare them.

## 2. Current Status of Research

Currently, high-frequency ultrasound and color Doppler ultrasonography have become important screening tools in breast cancer screening and clinical management. The sonographic presentation of breast cancer is based on pathological morphological changes. The diversity of pathological histology, gross staging, and immunohistochemical features of the breast cancer causes the sonographic presentation of breast cancer lesions to be complex and variable as well [5]. Especially, the early biological features and ultrasound manifestations of small breast masses are extremely atypical, or when early breast cancer masses do not show typical sonographic manifestations, they bring confusion to ultrasound diagnosis. In addition, traditional ultrasound elastography is a semiquantitative method to determine the hardness of lesions, and it is easily affected by physician subjectivity and manipulation during the operation. STE, compared with traditional elastography, obtains quantitative elastic modulus values, and it can quantitatively analyze the elasticity of soft tissues in real-time, which can effectively avoid the subjectivity of scoring methods and assess the elastic changes of the tissues by the changes of elastic modulus values [6]. It can effectively avoid the subjectivity of scoring methods and assess the elasticity changes of tissues by the changes of elastic modulus values and realize the study of tissue characterization. The quantitative display of tissue elasticity is obtained by the probe without applying pressure to the tissue, avoiding the influence of strain by the operator and/or the tissue, and under the same pressure, the soft tissue can produce different deformations according to its position and the position of the adjacent hard tissue. Shear waves are generated fully automatically by the probe, and the sweep technique is nondependent with repeatable image patterns and good repeatability of elastic modulus values [7].

Most of the studies on the differential diagnostic value of STE for benign and malignant breast lesions have been reported by scholars, and the methods are mostly based on surgical pathology as the gold standard for diagnosis [8]. The sensitivity of using the maximum elasticity reference value as the diagnostic threshold for benign and malignant lesions was higher than that of the average elasticity reference value, while the specificity of the former was lower than that of the latte. The application of the area under the ROC curve to compare the maximum and average elasticity values for the diagnosis of benign and malignant breast lesions showed that the accuracy of using the maximum elasticity value for the diagnosis of benign and malignant breast lesions was higher [9]. When the lesion is accompanied by hemorrhagic necrosis, calcification, or collagen fibrosis, elasticity measurement is performed [10].

Elastography, as a novel imaging technique that can reflect and measure tissue stiffness noninvasively, has gained widespread attention and rapid development among clinicians and sonographers not only to identify benign and malignant breast lesions but also to assess histological information by describing the distribution of internal tissue stiffness [11]. Eliminate cross-domain feature distribution differences in the feature space. After the source domain samples are migrated, the feature learning category prototype is obtained, and the training process of the feature classification model of the breast tumor pathological image in the target domain is guided based on this. Early elastography, such as strain force elastography, which requires external manual pressure to show elastic deformation based on tissue displacement, is highly operator-dependent, susceptible to external pressure, and poorly reproducible. In recent years, the current newer shear wave elastography technique acquires transverse wave signals in the tissues by ultrasound machines equipped with ultrafast imaging capture systems and calculates the shear wave velocity from the time difference between the adjacent peaks of the shear wave and the wavelength. Tissue stiffness can be quantitatively evaluated by the shear wave velocity, and this operation does not require operator pressure, overcoming the limitations of result variability and operator dependence.

## 3. Identification of Abnormal Ultrasound Breast Image Data Analysis Assisted by Shear Wave Elastography

### 3.1. Shear Wave Elastography-Assisted Ultrasound Breast Imaging Experiments

The ultrasonic radiation force comes from the change of linear momentum when the ultrasonic wave propagates in the medium, i.e., the ultrasonic wave in the medium will produce energy density difference because of absorption or scattering. Only in a viscoelastic liquid or solid with a certain attenuation coefficient can the sound radiation force be produced [12]. The action of acoustic radiation force by the emission of a series of detection pulses can get the corresponding position of the tissue vibration. The obtained vibration information for the relevant algorithm processing can get the displacement curve of the tissue. When the tissue is deformed because of the excitation, the echo signal of the same mass is detected with a certain time shift. The time-to-peak method is one of the most widely used methods to estimate the shear wave velocity using linear regression, which, firstly, determines the time of shear wave propagation to each detection point. Then, it makes a linear regression of each arrival time against the distance of the passage passed in the corresponding time and estimates the shear wave velocity from the slope of the linear regression. The shear wave velocity is estimated from the slope of the regression [13]. The variation of the vibration displacement with time for each of the *n* channels to the right of the acoustic radiation force excitation point can be represented. The slope of the mass point vibration displacement versus propagation time is fitted linearly by calculating the distance between the corresponding feature points and the time between wave propagation to the crest of the corresponding feature points to obtain the corresponding shear wave velocity value.

A total of 70 patients with 64 lumps suspected to be solid masses of BI-RADS grade 4 and above were collected from two hospitals, namely The Second Affiliated Hospital of Medical College of Zhejiang University and The Fourth Affiliated Hospital of Zhejiang University School of Medicine, without any treatment, and they were detected by routine ultrasonography and/or mammography of the breast. The above patients underwent multimodal ultrasound including 2D gray-scale, color Doppler with elastography for the masses suspected of BI-RADS grade 4 and above before undergoing pathological examination (hollow-core needle aspiration biopsy, minimally invasive episiotomy, mass excision, or radical surgery). The images were stored, and the data was recorded [14]. To improve diagnostic quality, the operating physician was trained in image acquisition and image quality control before the operation, and routine ultrasound and STE examinations were performed by a physician with 7 years of experience in breast ultrasound diagnosis using a high-quality line array probe from a fixed ultrasound instrument. The patient was placed in a supine position with arms raised to fully expose the breast, axilla, and upper and lower clavicle, and a routine radiographic scan was performed centered on the nipple. After finding the mass, the largest diameter section of the mass was selected, the probe was adjusted to clearly show the relationship between the mass and the surrounding tissues, and machine parameters such as depth, dynamic range, and depth gain compensation were adjusted to maintain the stability of the probe. To reduce the distribution difference between the domains at the category level, the feature distribution difference between the domains is often optimized and reduced by the MMD constraint on the average feature value of the entire domain. 2D gray-scale ultrasound images of the largest diameter section of the mass were acquired, and the mass size, margin, morphology, presence of lobulation and angulation, internal echogenicity, posterior echogenicity, and the presence of microcalcifications were recorded. The color flow signal within and around the mass was determined, and the PW mode was switched to obtain the spectral pattern and record the resistance index as shown in Table 1.

The study was performed by two physicians, one sonographer with 6 years of experience operating shear wave elastography and 20 years of experience operating conventional ultrasound practice, and the other with 6 years of experience operating conventional ultrasound practice and was trained to operate 30 cases of shear wave elastography on the ultrasound machine used in this study before the study began. The 30 cases of simulated training were not included in the data for this study. All ultrasound data were obtained using a Mindray ultrasound machine with a 14 L5 high-frequency line array probe (range 5–14 MHz). Each patient underwent a routine ultrasound examination before SWE. Before the examination, the patient was instructed to lie in a flat position with hands raised, and if the lateral breast was to be examined, the patient was turned slightly on his or her side to fully expose both breasts, and parameter settings such as gain and depth were adjusted according to the location and size of the breast mass. Then, the operator recorded basic information such as quadrant location, size, echogenicity, boundary, shape, and posterior echogenic attenuation of the breast lesion. Color Doppler flow imaging (CDFI) showed the peripheral and internal blood flow of the mass as shown in Figure 1.

The quantitative metrics for static-mode elastography and dynamic-mode elastography have an excellent interobserver agreement. The intragroup correlation coefficient ICC of dEmax in the dynamic mode is 0.962. The intragroup correlation coefficient ICC of dEmean in the dynamic mode is 0.915. The intragroup correlation coefficient ICC of DSD in the dynamic mode is 0.962. The interobserver agreement in the dynamic mode is slightly higher than that in the static mode.

Then, the Shear Wave real-time shear wave elastic ultrasound diagnostic instrument was used in two-dimensional gray-scale ultrasound mode to lightly place the probe on the skin. Determine the location of the breast lesion, add a sufficient amount of coupling agent, and fix the probe without applying pressure. Then, switch to SWE mode, place the elastic sampling frame in the area of interest, adjust the size of the real-time elastic imaging area, ask the patient to hold his breath if necessary, and rest for about 3 s [15]. If necessary, the patient was instructed to hold his breath, and the image was stored in a fixed frame after standing for approximately 3 s to 5 s to stabilize. Then, the same area of interest was positioned three times, the maximum elastic modulus value (*E*_max_) and the average elastic modulus value (Eman) of the shear wave were measured, and the average value of Emax and Eman of the three groups was taken as the final data. The dynamic changes of the elastic modulus value of the area of interest were continuously observed, and the maximum and minimum changes of Emax were taken to obtain the extreme difference of the change of *E*_max_. There is a 90° phase difference between stress, and hence, the ideal viscous body is represented by a viscous pot, which means that the container contains a liquid that obeys Newton's law of fluid. Compare the elastic modulus values of each group as shown in Figure 2.

A review of the relevant literature and the results of the early STE pretest in this study suggest that compared with benign lesions, malignant solid lesions have a “multivariable sign” with variable and unstable elastic signals, a “hard ring sign” with high surrounding elastic modulus values, and a “black hole sign” with the absence of internal shear wave elastic signals. Therefore, in this study, we prospectively performed a comprehensive analysis of lesions based on the presence or absence of these three features, readjusted the first BI-RADS classification, and compared the diagnostic efficacy of the two examination methods using pathological findings as to the gold standard [16]. This section covers standard heterogeneous mimic elasticity measurements based on an ultrasound data acquisition platform to compare focused versus unfocused comb pulse excitation modalities at different parameters. Hypotheses are formulated from the results of the first set of standard heterogeneous mimic body pre-experiments. Hypothesis one is verified by observing the acoustic field energy distribution under focused and unfocused comb pulse excitation methods by linear and convex arrays comb excitation pulse simulation. The proposed hypotheses one and two are verified by the second set of standard mimic experiments, and finally, the excitation algorithm used in this study is selected.

The midpoint of the probe was aligned with the marker point. The long axis of the probe was parallel to the muscle fibers. No pressure was applied. The muscle echogenicity and muscle fiber direction were carefully observed on the grayscale image. After displaying more than 3 continuous muscle fiberss, the shear wave elastography mode under the elastography menu was selected, the left and right borders of the region of interest (ROI) were adjusted to the maximum, and the upper and lower boundaries of the ROI are extracted. The patient was asked to hold his breath, the elastography image was acquired. For the upper right corner, the corner motion stability index (M-STB index) of the image was five green stars. Ten subjects were randomly selected, and the control group measured the trapezius muscle from the spinous process of the seventh cervical vertebra to the midpoint of the left acromion line. The case group measured the trapezius trigger point area from the spinous process of the seventh cervical vertebra to the midpoint of the acromion line on the painful side, and the mean values of SWVmax, swVmean, and SWVmin were recorded three times. The labeling of skin lesion images often requires experienced doctors or experts in the field to complete, and the labeling cost is much more expensive than natural visual images. The subjects were tested by 2 physicians separately (without knowledge of each other's findings and knowledge of the patient's pain level) according to the above measurements, and the reproducibility of the measurements between the different tests was compared. Physician A measured the same subject again half an hour later to compare the reproducibility of measurements between the times for the same examiner.

### 3.2. Discriminatory Analysis of Abnormal Data from Glandular Images

The prototype network model introduces the idea of a statistical generative model that learns a generative model about a dataset by extending the variational self-encoder rather than using independent sample points as the learning object. The main module of the model, namely the statistical network, summarizes a series of data sample points into a statistical vector [17].

(1) $$\begin{array}{c} \mu_{c}=\frac{1}{\left|\varsigma_{c}\right|}\sum_{x_{i}\in S_{c}}f\left(x_{i}^{2},\theta^{2}\right). \end{array}$$

In this case, the direct migration of trained classification models to new datasets inevitably results in a large degree of loss of effectiveness. Also, the new dataset faces the problem of labeling difficulties. From the above, PTGAN aims to achieve the migration of the model trained in the source domain data to the unlabeled target domain without labeling the new data to improve the classification of breast tumor pathology images. Firstly, a dataset of the breast tumor images with existing labels in the source domain is defined, and a dataset of unlabeled target breast tumor images to be classified is defined as the target domain. It represents the number of samples in the source and target domains, respectively, representing the class labels of the samples in the source domain.

(2) $$\begin{array}{c} h_{i}^{s}=f\left(x_{i}^{s},\theta_{f}^{2}\right),\\ h_{j}^{t}=f\left(x_{j}^{t},\theta_{f}^{2}\right). \end{array}$$

After the target-biased generation of adversarial networks, the migration effect of the samples in the source and target domains at the image style level is guaranteed. However, the migration problem at the feature level in the classification task has not been solved. Therefore, this subsection designs a prototype migration module to further migrate the features extracted from the network by cross-domain feature migration loss to eliminate the differences in cross-domain feature distribution in the feature space. It is the site where most breast diseases occur. Masses in the breast are common clinical manifestations of breast diseases, most of which are caused by benign diseases, such as fibroadenoma, cysts, etc. The source domain samples are migrated to obtain the feature learning category prototype, and this is used to guide the training process of the feature classification model for breast tumor pathology images in the target domain as shown in Figure 3.

MMD is the maximized mean deviation used to measure the difference in data distribution between the source and target domains. After the MMD loss constraint, the difference between the distribution of the source domain features and the target domain features after style transformation is reduced, and domain adaptation is achieved at the feature level.

(3) $$\begin{array}{c} L_{MMN}=\left\|\frac{1}{N_{s}}\sum_{i=1}^{N_{s}}h_{i}^{s}+\frac{1}{N_{s}}\sum_{j=1}^{N_{t}}h_{j}^{s}\right\|,\\ D_{KL}\left(p\|q\right)=\sum_{c=1}^{c}\ln\frac{p_{i}^{c}}{q_{j}^{c}}. \end{array}$$

As shown in Figure 4, often in viscoelastic studies of biological tissues, some biological models are used to fit the mechanical properties of the tissues [18]. For purely viscous materials, there is a 90° phase difference between stress. Hence, the ideal viscous body is represented by a vicious pot, representing a container containing a liquid obeying Newton's law of fluids. However, for purely elastic materials, there is no phase difference between stress. Hence, the ideal elastomer is represented by a spring [19]. The Voigt model for the study of bio-viscoelasticity can be obtained by connecting the spring in parallel with the viscous pot. To improve the performance of deep neural networks during medical image classification, it is common to consider scaling up the model training by increasing the amount of labeled medical image data.

However, in real scenarios, these medical data differ to some extent in terms of light intensity, viewpoint, background, etc. Meanwhile, the quality of medical image annotation relies on the degree of expertise of the annotators, which requires years of accumulated expertise and experience [20]. Provide information, including tumor size, shape, edge, echo pattern, whether there is attenuation behind, and whether there is calcification inside, etc., to provide a basis for finding breast cancer. With the increasing standard of intelligent-assisted classification and diagnosis of skin lesion images in clinical practice, the annotation of skin lesion images often requires experienced doctors or experts in the field to complete, and its annotation cost is much more expensive compared with natural visual images. Thus, the task of automatic classification of skin lesion images faces difficulties and limitations, such as complex sample data, uneven distribution, and expensive annotation of labeled samples.

Existing research works mainly focused on the fields of machine learning and data mining, which can be summarized into two categories: clustering and domain adaptive methods. These research works assume that the number of classes of the target medical image is known in advance and then applied to the image classification problem lacking labeled information to achieve unsupervised medical image classification results. However, this assumption premise is usually difficult to hold in practical scenarios because, in medical images, there will be additional unexpectedly generated symptom classes in addition to the already known symptom classes, a situation that existing clustering and domain adaptive algorithms cannot cope with. In other words, the existing machine learning clustering algorithms cannot automatically construct information about the categories of the data and cannot interpret conceptual information about the categories of objects, etc., without external supervision.

## 4. Analysis of Results

### 4.1. Experimental Results

Benign masses such as breast adenopathy and fibroadenoma have loosely arranged tumor cells with a high content of interstitial mucopolysaccharides, and therefore, lower hardness values. In contrast, malignant tumors contain abundant connective tissues, blood vessels, and lymphatic vessels inside, and the tumor cells are tightly wrapped by proliferative fibrous tissues. In addition, malignant tumors have the ability of distant invasion, and during the process of tumor growth, they continuously adhere to and invade the surrounding tissues, resulting in adhesions between the masses and the surrounding tissues, thus reducing the elasticity of the tissues leading to an increase in the hardness value. Class 4A masses were corrected to class 3, of which 2 cases were missed. 1 case was ductal carcinoma in situ and the other case was ductal carcinoma in situ with acne-like necrosis 4 masses were upgraded from category 4A to category 4B, 1 of which was correctly upgraded, and the pathology was intraductal papillary carcinoma, while the remaining 3 masses were benign, namely, lobular granulomatous mastitis, adenopathy with fibroadenoma formation, and focal chronic inflammatory cell infiltration, all of which were large. Six masses were downgraded from category 4B to 4A, three of which were intraductal papilloma's and were correctly downgraded, while the other three were incorrectly downgraded, with the diameters of 11 mm, 5 mm, and 11 mm, respectively, and the pathological types of intraductal carcinoma, ductal carcinoma in situ, and ductal carcinoma in situ with local infiltration, respectively. It also has important clinical value in the differential diagnosis of benign and malignant breast lesions. However, the ultrasound charts of benign breast lesions and breast cancer now overlap to a certain extent. It is also complicated and changeable because of the diversity of its clinicopathological characteristics. The ratio, SD, and Emax of all three masses were below the diagnostic threshold, as shown in Figure 5.

Breast cancer is usually insidious, with no clinical symptoms in the early stage and is usually detected by chance. Routine ultrasound screening for breast cancer has the advantages of noninvasiveness, nonradiation, low price, and good reproducibility. Together with mammography and magnetic resonance imaging, it has become the three major imaging methods for noninvasive diagnosis of breast diseases.

To standardize the description of breast masses, the US-BI-RADS classification criteria are gradually applied in clinical practice. Although the sensitivity of US-BI-RADS was fair, the specificity, accuracy, and NPV were low, and the benign rate was as high as 51% in grade 4 and above masses enrolled in this study. It can overcome the interference of tissues outside the region of interest, has high repeatability, and has unique advantages in the diagnosis and differential diagnosis of breast diseases. Therefore, it can overcome the subjective influence and inherent defects of stress elastography technology. If such patients were blindly selected for puncture biopsy or surgical management, it would not only cause trauma to the patients but also result in a waste of valuable medical resources. In addition, the mid- and long-term follow-up of conservative treatment of benign masses confirmed by puncture biopsy faces the challenge of whether to rashly downgrade the mass to benign based on the previous pathological findings or to determine whether the mass has undergone minor suspicious changes based on the morphological features of the mass, which poses a certain challenge to ultrasonographers at each follow-up visit. In addition, it is difficult to use puncture biopsy as a routine follow-up in clinical practice. Therefore, there is an urgent need for a safe, reliable, and simple noninvasive method as a supplement to US-BI-RADS to improve the specificity and accuracy of diagnosis to reduce unnecessary puncture biopsies and surgical management as shown in Figure 6.

Neovascularization is an important stage in the growth of malignant masses over 2–3 mm, and tumor growth and metastasis are associated with angiogenesis, which is a hot topic for research into new anticancer approaches. Many antineovascularization therapies use this principle to destroy or limit tumor angiogenesis. The current study demonstrates the relationship between breast malignant mass stiffness and blood flow, while shear wave elastography is easy and less time-consuming to perform compared to ultrasonography. Without the need for intravenous injection and background software analysis, it allows for a rapid understanding of the approximate fibrous tissue and blood flow within the mass and assessment of the sensitivity of ant neovascular therapy. A higher-quality image can be obtained on static mode elastography, three levels of frame rate can be selected in dynamic mode elastography, and multiple images can be selected in succession. Firstly, the sample size of this study was not large enough. A total of 70 breast masses were included in this study, including 64 malignant masses. The sample size should be expanded for further study in future studies. Secondly, in the quantitative analysis of breast lumps, the ROI should be sampled several times to determine the quantitative indicators and averaged to make it more objective. Thirdly, the choice of ROI location also affects the perfusion of the time-intensity curve. Angiogenesis is more active in the peripheral region of a malignant mass than in the central region. The central region is filled with bridging and fibrous tissue. Hence, the parenchyma is stiffer, and vascular growth is difficult in it. Hence, the interior is not as vascular, and again, there is central calcified necrosis formation.

### 4.2. Results of Anomalous Data Identification

To improve the automatic classification performance of breast tumor histopathology images with insufficient labeled samples, semisupervised learning has been gradually introduced in the field of medical image classification research. Compared with unsupervised learning, the semisupervised learning approach can apply the inherent characteristics and patterns of the unlabeled sample data and can improve the status quo of unsupervised learning classification methods with unsatisfactory results accuracy. Therefore, this chapter introduces a semisupervised framework for classifying histopathological images of breast tumors. It utilizes a small number of labeled samples and many unlabeled samples to constitute the training data, effectively overcoming the overfitting problem of unsupervised classification methods and improving the classification accuracy without the need for a large-scale data annotation effort. The PTGAN model was used to test the classification performance on the breast tumor pathology image dataset while reporting the performance of multiple breast tumor pathology image classification methods used on the BreaKHis dataset. The experimental results of this method on image samples with different magnifications are shown in Table 2.

The source domain image samples do not have any overlapping data with the target domain image samples. In addition, considering the different relevance of sample data in different source domains for migration to the target domain, a fuzzy attention mechanism is designed in this chapter to calculate their weights for migration to the target domain. This method, firstly, determines the time for the shear wave to propagate to each detection point. Then, it performs a linear regression on the distance between each arrival time and the passage through the corresponding time and estimates the speed of the shear wave from the slope of the linear regression. With the learned weights of different source domains, MFAN can learn a shared robust feature space for breast tumor histopathology images and train the fine-tuned classification models adapted to the target domain by label inference.

Most of the available research works report classification results in two categories, benign and malignant. This chapter focuses on the problem of dichotomizing PTGAN in breast tumor pathology images, and therefore, it only considers the experimental results of existing work under the dichotomization task at the image level for control. The experiments of the existing work are performed at 40x, 100x, 200x, and 400x magnifications for binary classification and multiclassification problems. Based on the BreaKHis dataset, an 85% accuracy at the patient level was obtained by applying different features. AlexNet is used to conduct a two-classification study on pathological images of breast tumors. The average accuracy rate of the image level is 89.0%, and the average accuracy rate of the patient level is 90.0%. To demonstrate the variation of loss versus accuracy on the training and test sets during PTGAN training, this subsection shows the accuracy and the curve dynamics of network loss during the model training iterations in Figure 7 using 100x magnification breast tumor pathology image data as an example.

The style migration across domains is achieved by the target domain bias-generative adversarial network to reduce the style differences between source and target domains. The extracted sample features are mapped into a cross-domain feature space by cross-domain loss constraints, thus training the classification in the cross-domain feature space using source and target domain features. To improve the quality of diagnosis, the operating doctor conducts image acquisition training and image quality control before the operation. Routine ultrasound and SWE examinations are completed by a doctor with 7 years of breast ultrasound diagnosis experience using a high-quality linear array probe with a fixed ultrasound instrument. Validation tests are conducted on the BreaKHis dataset, and the core module of PTGAN is discussed in this chapter, showing that it has excellent feature extraction capabilities. Also, it achieves an accuracy level closer to that of supervised learning methods without the advantage of large-scale data annotation efforts, and it scales well.

## 5. Conclusion

Shear wave elastography may provide a certain reference basis for the selection of breast cancer treatment strategy and prognosis judgment. To determine the accuracy of TDPM measurement, a total of four gelatin body molds with different agar contents were made as validation objects in this experiment, and the body molds were soaked in glycerol to increase their toughness. SWE and mechanical tensile experiments were performed. The conventional SPM was introduced to compare the results of the two ultrasonic measurements, and the results of the mechanical tests were used as the gold standard to verify the results of the ultrasonic experiments. The results show that the displacement data measured by SPM are not well-fitted linearly in the process of fitting the group velocity. However, TDPM is more accurate in detecting the feature points because of the improved sampling resolution. The linear fit is better, and the fitted shear wave group velocity is more accurate. The measurement results of TDPM have less variance, less random error, better precision, and are closer to MT results. Because of the complex pathological process of adenopathy and the lack of specific sonographic features, there is some overlap with the sonogram of breast malignancy, and the misdiagnosis rate is high. In clinical practice, we should fully understand the ultrasound image features and pathological characteristics of adenopathy, combine clinical data, image features, and elastography parameters to make a comprehensive analysis. When suspicious signs are found, puncture biopsy under ultrasound guidance promptly to improve the diagnostic compliance rate and reduce the misdiagnosis rate.

## Figures and Tables

**Figure 1:** Interobserver agreement of quantitative metrics for shear fluctuation/static mode elastography.

**Figure 2:** Experimental steps.

**Figure 3:** Migration metric learning framework diagram.

**Figure 4:** Radon transformation method for shear wave group velocity.

**Figure 5:** ROC curves for the diagnosis of breast masses.

**Figure 6:** Relationship between quantitative indicators of shear wave static mode elastography and quantitative indicators of ultrasonography in benign masses.

**Figure 7:** Accuracy and loss variation on the test and training sets.

**Table 1:** Types of pathology studied by shear wave.

Malignant mass	Number of cases	Benign mass	Number of cases
Invasive ductal carcinoma	2	Fibroadenoma	3
Ductal carcinoma in situ	4	Adenopathy	4
Papillary carcinoma	10	Papilloma	11
Mucinous carcinoma	20	Benign phyllodes tumor	24
Invasive lobular carcinoma	10	Adenopathy with papilloma	10
Invasive adenocarcinoma	18	Interstitial sclerosis	18
Total	64	Total	70

**Table 2:** Image classification results of PTGAN model on BreakHis dataset.

Multiple	Accuracy 1	Accuracy 2	Recall rate	F1-score
40x	84.9	94.6	89.3	88.5
100x	88.9	93.4	88.7	97.5
200x	90.5	96.9	80.6	95.1
400x	84.3	86.3	95.5	80.8
Average value	83.4	89.5	87.8	95.5

## Data Availability

The data used to support the findings of this study are available from the corresponding author upon request.
